# Data Feature Extraction Method of Wearable Sensor Based on Convolutional Neural Network

**DOI:** 10.1155/2022/1580134

**Published:** 2022-01-25

**Authors:** Baoying Wang

**Affiliations:** College of Electronics and Internet of Things, Chongqing College of Electronic Engineering, Chongqing 401331, China

## Abstract

With the rapid development of society and science technology, human health issues have attracted much attention due to wearable devices' ability to provide high-quality sports, health, and activity monitoring services. This paper proposes a method for feature extraction of wearable sensor data based on a convolutional neural network (CNN). First, it uses the Kalman filter to fuse the data to obtain a preliminary state estimation, and then it uses CNN to recognize human behavior, thereby obtaining the corresponding behavior set. Moreover, this paper conducts experiments on 5 datasets. The experimental results show that the method in this paper extracts data features at multiple scales while fully maintaining data independence, can effectively extract corresponding feature data, and has strong generalization ability, which can adapt to different learning tasks.

## 1. Introduction

Wearable devices are smart devices that can be installed on people, animals, and objects, and can sense, transmit, and process information [1]. Sensors are the core carrier, and wearable sensors are an extension of human senses. With the rapid development of the Internet of everything and society, human health issues have also received widespread attention. Various health indicators and parameters of the human body can also be connected to the Internet for monitoring and analysis. Perceive human behavior through wearable sensors, which can be used in medical health, sports fitness, disease prevention, and treatment, especially in the daily monitoring of elderly people [2–8]. With the intelligent development of wearable devices, sensors such as accelerometers, magnetometers, and heart rate meters are built into smartphones and smart bracelets [9]. The sensors can continuously track and collect human behavior data, fully protecting personal privacy as well. Users only need to wear their mobile phones or smart bracelet to complete data collection.

Most of the data collected by wearable sensors are sequence data. Currently, models based on recurrent neural networks (RNN) and convolutional neural networks (CNN) are mainly used to predict and identify sequence data [10, 11]. Although the accuracy of the RNN-based data prediction and recognition model is slightly higher than the accuracy of the CNN-based model, the cyclic nature and data-dependent characteristics of the RNN model make it difficult to achieve high parallelization on the edge side, which leads to low computing efficiency on the edge hardware platform. CNN can achieve higher computational parallelism and higher applicability. Therefore, this paper uses a CNN-based model to extract the data features of wearable sensors and perform human behavior recognition [12, 13].

## 2. Related Work

Figure 1 shows the process of feature extraction of wearable device sensing data and the output results based on CNN. First, the human body's acceleration, heart rate, and other data are collected through the sensor in the wearable device, and the original data is scanned with a fixed time window to obtain samples as the input of the CNN model. Then, the model is used to identify its specific behavior category. After obtaining each behavior category, an individual behavior dataset is generated.

### 2.1. Wearable Sensors and Data Collection

Wearable devices first appeared in the middle of the 20th century. The traditional method is to place sensors directly on the user to collect user motion data. The sensors used in data acquisition equipment mainly include accelerometers, gyroscopes, magnetometers, smartphones, barometers, pressure sensors, and EMG signal detectors, among which accelerometers and gyroscopes are more common. The accelerometer mainly measures the force of the device and can sense acceleration in any direction; the gyroscope judges the current movement state of the device through its rotation state (angle and angular velocity). With the development of smart devices, researchers generally design embed sensors in mobile devices. Chacon et al. designed a new pulse oximeter by embedding sensors in portable medical equipment, providing real-time monitoring of the physical condition of the elderly [14]. For the feature extraction of wearable sensor data, complex behaviors in general life can be expressed through various basic action combinations. For example, eating snacks includes several basic actions such as holding and eating.

Gu et al. introduced the emerging pattern to describe the discriminative pattern of significant changes between data categories and identified sequential, interlaced, and concurrent activities in a unified framework, thereby identifying sensor features and classifying activities [15]. Wang et al. proposed a hierarchical recognition method to infer ongoing activities in a multistage process to better distinguish similar activities and improve overall performance [16]. In terms of complex behavior recognition, Chang et al. considered the interaction between people and the surrounding environment using sensors distributed on people and objects to collect behavioral data, which improves the extraction of data features of complex behaviors [17].

### 2.2. Data Feature Extraction

In human behavior recognition, the most representative algorithm is the improved dense trajectories (IDT) algorithm [11]. It is a dense optical flow trajectory algorithm based on dense trajectories (DT). Before CNN was applied, IDT was the best algorithm for human behavior recognition. With the development of CNN, Ye et al. proposed the two-stream method to extract behavioral features in video space and time. Compared with IDT, the two-stream method is more robust [18]. The convolutional 3D method proposed by Torfi et al. can directly process video [19]. The effect is very good in spatiotemporal feature extraction. This method effectively improves the recognition speed, but the accuracy is low. Jin et al. put forward the time-sensitive network (TSN) method [20]. By segmenting the long video, the problem of the inability to model the long-term structure in the two-stream method is solved, but the TSN method has a complex structure. The recognition speed is slow. Wu et al. discussed the deep local video feature (DLVF) method based on the TSN method, assigning different weights to different segments in TSN and fusing the judgment results of different segments more reasonably [21]. Chanti et al. envisioned a behavior recognition method based on temporal and spatial weighted gesture motion characteristics through dynamic time warping and Fourier time pyramid algorithm modeling, and finally improved the accuracy of human behavior recognition [22].

## 3. Wearable Sensor Data Feature Extraction Method Based on CNN

The data feature extraction studied in this paper is suitable for sensors installed on people, animals, and objects, but the sensors must move with the appendages so that the relevant data features can be extracted, and their behaviors can be analyzed to obtain a behavior set. For example, when a person is running, their running behavior is recognized through the data characteristics of parameters such as legs, hands, and heart rate.

For the extraction of wearable sensor data features, the acceleration data, angular velocity data, and magnetic field data output by the wearable sensor are first fused by the extended Kalman filter fusion algorithm. Then, the preliminary state estimation of the human behavior represented by the wearable sensor output data is obtained, and the CNN model is used to process the collected data in parallel to get the result of human behavior recognition.

### 3.1. Data Fusion

At present, the commonly used human behavior data feature decomposition methods are estimation methods based on Kalman filtering, which mainly include unscented Kalman filtering, extended Kalman filtering, and volume Kalman filtering [23]. The estimation methods based on non-Kalman filtering include the complimentary filtering algorithm and the gradient descent algorithm. Through the comparison of several methods, this paper selects the extended Kalman filter method to identify the behavior of the sensor.

The Kalman filter is an algorithm designed for linear systems at the beginning of its design and cannot be applied to nonlinear systems, but in practice, most systems are nonlinear, and it is impossible to directly use the Kalman filter to solve nonlinear systems. In response to this problem, scholars began to transform the Kalman filter to improve and optimize its performance so that it can be applied to nonlinear systems. In this process, an extension of the Kalman filter to nonlinear systems has been produced.

This paper uses the data fusion algorithm based on the extended Kalman filter to realize the human behavior recognition capability of the inertial sensor.  Figure 2 shows the specific implementation process of the data fusion algorithm based on the extended Kalman filter. As shown in the figure, the system has three different types of input data. The gyro data is measured in deg/s, and the angular velocity is measured on three axes. The accelerometer data measures acceleration in *g*. The magnetometer data measures the magnetic field in Gaussian units. The gyro data is used as an input to update the prior state estimation. At the same time, the accelerometer and magnetometer data are used as a fixed reference to correct the error in the prior state estimation. The following is the specific implementation process of this method.

In the data fusion algorithm based on the extended Kalman filter, it is defined that {*n*} represents the navigation coordinate system and {*b*} represents the sensor coordinate system. First, the initial Euler angle is calculated using the accelerometer and magnetometer data acquired at the initial moment. The initial pitch angle *x*_0_ and the initial roll angle *y*_0_ are obtained from the acceleration data, and the initial yaw angle *z*_0_ is obtained from the magnetic field data which are as follows:

(1) $$\begin{array}{c} x_{0}=\arcsin\frac{a_{y}}{\sqrt{a_{x}^{2}+a_{y}^{2}+a_{z}^{2}}},\\ y_{0}=\arctan\frac{-a_{x}}{a_{z}},\\ z_{0}=\arctan\frac{m_{x}\cos\left(y_{0}\right)+m_{b}\sin\left(y_{0}\right)}{m_{x}\sin\left(y_{0}\right)\sin\left(x_{0}\right)+m_{y}\cos\left(x_{0}\right)-m_{z}\cos\left(y_{0}\right)\sin\left(x_{0}\right)}, \end{array}$$

where *a*_*k*_=[*a*_*x*_, *a*_*y*_, *a*_*z*_]^*T*^ defines the acceleration data at the initial moment, and *m*_*k*_=[*m*_*x*_, *m*_*y*_, *m*_*z*_]^*T*^ presents the magnetic field data at the initial moment. Through the conversion between the Euler angle and a quaternion, the quaternion of the initial moment state can be obtained.

The quaternion is a four-dimensional vector that can express various poses in space without any singularity. The posture represented by the quaternion can be understood as a coordinate system rotated by another coordinate system. Then, the final coordinate relative to the original coordinate can be regarded as a rotation of the original coordinate, assuming that the angle of rotation is *θ*, $K={\left[\begin{array}{ccc} k_{x} & k_{y} & k_{z} \end{array}\right]}^{T}$ represents the equivalent rotation axis, then $q={\left[\begin{array}{cccc} q_{0} & q_{1} & q_{2} & q_{3} \end{array}\right]}^{T}={\left[\begin{array}{cccc} \cos\theta /2 & k_{x}\sin\theta /2 & k_{y}\sin\theta /2 & k_{z}\sin\theta /2 \end{array}\right]}^{T}$ and *q*_0_^2^+*q*_1_^2^+*q*_2_^2^+*q*_3_^2^=1. The state transition equation in the continuous domain mainly uses quaternion differential equations, which can be defined as follows:

(2) $$\begin{array}{c} \dot{q}=\frac{1}{2}\Omega \left(\omega_{t}\right)q, \end{array}$$

where $\dot{q}$ represents the differential of the quaternion, *Ω*(*ω*_*t*_) is the rotation matrix derived from the nature of the quaternion, expressed by the angular velocity data *ω*_*t*_=[*ω*_*x*_, *ω*_*y*_, *ω*_*t*_]^*T*^ measured by the gyroscope at the time *t* and has the following form:

(3) $$\begin{array}{c} \Omega \left(\omega_{t}\right)=\left[\begin{array}{cccc} 0 & -\omega_{x} & -\omega_{y} & -\omega_{z}\\ \omega_{x} & 0 & \omega_{z} & -\omega_{y}\\ \omega_{y} & -\omega_{z} & 0 & \omega_{x}\\ \omega_{z} & \omega_{y} & -\omega_{x} & 0 \end{array}\right]. \end{array}$$

The application field of the Kalman filter is the discrete domain. For this reason, it is necessary to convert the quaternion differential equation in the continuous domain into the discrete domain. By displaying the derivation, the continuous-time system can be rewritten as follows:

(4) $$\begin{array}{c} \dot{q}=\lim_{T⟶0}\frac{q\left(t+T\right)-q\left(t\right)}{T}\\ =\frac{1}{2}\Omega \left(\omega_{t}\right)q\left(t\right). \end{array}$$

To transform this equation into a discrete-time equation, the time step *T* between each execution of the algorithm is used in the digital system. In this way, we can know the following:

(5) $$\begin{array}{c} q\left(t+T\right)=q\left(t\right)+\frac{1}{2}\Omega \left(\omega_{t}\right)q\left(t\right)T\\ =\left(I+\frac{1}{2}\Omega \left(\omega_{t}\right)T\right)q\left(t\right). \end{array}$$

Because the bias of the gyroscope is also considered in the system, this paper defines the state vector of the system as a unit quaternion and gyroscope bias. The update equation of the state vector can be obtained through the abovementioned analysis, which is as follows:

(6) $$\begin{array}{c} \left[\begin{array}{c} q_{t+1}^{-}\\ \omega_{bt+1} \end{array}\right]=\Phi_{t}•\left[\begin{array}{c} q_{t}\\ \omega_{bt} \end{array}\right], \end{array}$$

where *q*_*t*_ is the optimal estimated value of the quaternion of the unit behavior at the previous moment, *q*_*t*+1_^−^ is the suboptimal estimated value of the quaternion of the unit behavior at the current moment, and Φ_*t*_ is the state transition matrix. The specific expression is as follows:

(7) $$\begin{array}{c} \Phi_{t}=\left[\begin{array}{cc} I_{4\times 4}+\frac{T}{2}\Omega \left(\omega_{t}\right) & 0\\ 0 & I_{3\times 3} \end{array}\right]. \end{array}$$

The quaternion norm is not retained in the state equation. Since the angular position can only be correctly represented by a unit quaternion, it is necessary to introduce a normalization unit to ensure the integrity of the data.

The Jacobian matrix of the state transition equation is solved as follows:

(8) $$\begin{array}{c} G_{t}=\frac{\partial \left[q_{t+1}/\omega_{bt+1}\right]}{\partial \left[q_{t}/\omega_{bt}\right]}. \end{array}$$

It is solved by assuming that the noise between each axis of the accelerometer, gyroscope, and magnetometer is independent of each other. In this system, the state transition matrix that the system relies on is described by the gyroscope data, so the process noise covariance matrix directly depends on the gyroscope. In the measurement model, the measurement noise comes from the noise of the accelerometer and magnetometer. Therefore, the process noise covariance matrix *Q*_*t*_ and the measurement noise covariance matrix *R*_*t*_ can be determined as follows:

(9) $$\begin{array}{c} Q_{t}=\left[\begin{array}{cc} \omega_{n} & 0\\ 0 & \omega_{\text{bn}} \end{array}\right],\\ R_{t}=\left[\begin{array}{cc} a_{n} & 0\\ 0 & m_{n} \end{array}\right]. \end{array}$$

In the abovementioned formula, *ω*_*n*_ is the gyroscope measurement noise, *ω*_*bn*_ is the gyroscope bias noise, *a*_*n*_ is the accelerometer measurement noise, and *m*_*n*_ is the magnetometer measurement noise.

Therefore, the prior error covariance at time *t* can be further solved as follows:

(10) $$\begin{array}{c} P_{t}^{-}=G_{t}P_{t-1}G_{t}^{T}+Q_{t-1}. \end{array}$$

*P*_*t*−1_ represents the posterior error covariance matrix of the previous filter iteration. The behavioral state quaternion obtained by (6) is calculated from the output data of the gyroscope and the optimal behavioral state at the previous moment. It is the behavior obtained during the long-term operation by relying only on the output of the gyroscope. The state is not reliable, so it is necessary to fuse the accelerometer and magnetometer data to modify the state to obtain the final optimal behavior.

To calculate the measurement equation of the magnetometer, first convert the magnetic field data from the sensor coordinate system to the navigation coordinate system to obtain the magnetic field data in the navigation coordinate system. *m*^*b*^ represents the magnetic field data in the sensor coordinate system, and *m*^*n*^ represents the magnetic field data in the navigation coordinate system, which are as follows:

(11) $$\begin{array}{c} \left[\begin{array}{c} 0\\ m_{x}^{n}\\ m_{y}^{n}\\ m_{z}^{n} \end{array}\right]=q_{t}^{-}⊗\left[\begin{array}{c} 0\\ m_{x}^{b}\\ m_{y}^{b}\\ m_{z}^{b} \end{array}\right]⊗{\left(q_{t}^{-}\right)}^{•}. \end{array}$$

In the measurement model, it is assumed that the magnetic field in the navigation coordinate system has no data in the east direction and only in the north and sky directions. After the magnetic field data is processed and then converted to the carrier coordinate system, the measured value ${\bar{m}}_{b}$ of the magnetic field strength can be obtained, which is as follows:

(12) $$\begin{array}{c} {\bar{m}}_{b}={\left(R_{b}^{n}\right)}^{-}\left[\begin{array}{c} 0\\ \sqrt{m_{x}^{n}\times m_{x}^{n}+m_{y}^{n}\times m_{y}^{n}}\\ m_{z}^{n} \end{array}\right]. \end{array}$$

The measurement equation of the accelerometer is calculated. In the navigation coordinate system, the reference direction of the gravity field is $g={\left[\begin{array}{ccc} 0 & 0 & 1 \end{array}\right]}^{T}$, and the measured value of acceleration ${\bar{a}}_{b}$ is obtained from the equation:

(13) $$\begin{array}{c} {\bar{a}}_{b}={\left(R_{b}^{n}\right)}^{-}\cdot g. \end{array}$$

The obtained magnetic field data and acceleration data are normalized, and the processed data is denoted as *Z*_*t*_. Finally, the total measurement equation can be obtained from the following equation:

(14) $$\begin{array}{c} h_{t}\left(q_{t}^{-}\right)=\left[\begin{array}{c} {\bar{a}}_{b}\\ {\bar{m}}_{b} \end{array}\right]. \end{array}$$

The Jacobian matrix of the measurement equation is calculated as follows:

(15) $$\begin{array}{c} H_{t}=\frac{\partial h_{t}\left(q_{t}^{-}\right)}{\partial \left(q_{t}^{-}\right)}. \end{array}$$

Through the calculated prior error covariance, the Jacobian matrix of the measurement equation, and the measurement noise covariance matrix, the Kalman gain can be calculated as follows:

(16) $$\begin{array}{c} K_{t}=P_{t}^{-}H_{t}^{T}{\left(H_{t}P_{t}^{-}H_{t}^{T}+R_{t}\right)}^{-1}. \end{array}$$

The posterior error covariance matrix is updated, which is as follows:

(17) $$\begin{array}{c} P_{t}=\left(I-K_{t}H_{t}\right)P_{t}^{-}. \end{array}$$

Finally, a more accurate posterior state estimate can be obtained, which is as follows:

(18) $$\begin{array}{c} q_{{}_{t}}=q_{t}^{-}+K_{t}\left(Z_{t}-h_{t}\left(q_{t}^{-}\right)\right). \end{array}$$

### 3.2. Feature Extraction of Sensor Data Based on CNN

The basic calculation process of the CNN designed in this paper is shown in Figure 3, where *N* pairs of feature data are taken and weight parameters are considered as input. The corresponding *N* pairs of data are multiplied, and then the *N* results of the multiplication are accumulated.

Convolution calculation is the largest calculation part of the CNN model. To improve the computational efficiency of convolution calculations, this paper uses multiple channels and multiple filters to perform calculations in parallel. The specific process is shown in Figure 4. In the figure, the input feature data size is *H*_in_ × *W*_in_, the convolution kernel size is *K*_*x*_ × *K*_*y*_, the input channel is CH_in_, the number of convolution kernels is *K*, and *N* is the channel parallelism.

Multichannel parallelism cuts the feature data and each weight data into multiple sub-blocks along the input direction. The input channel dimension of each sub-block is *N*, and *N* corresponding data is taken out from the feature data sub-block and weight sub-block, respectively. Multifilter parallelism is the simultaneous calculation of input weights and multiple convolution kernels. Figure 4 shows the process of the sub-block convolution operation. The specific calculation process is as follows:

1. As shown in Figure 4(a), the feature data and the first data in the *n* channel directions of the 2 convolution kernels are taken out at the same time, and the corresponding data taken out respectively are multiplied, then accumulated in the channel direction, and the result is output.
2. As shown in Figure 4(b), the weight remains unchanged, and the feature data is slipped, so that the first data on the *N* channels of the weight is multiplied by part of the feature data and accumulated in the direction of the channel.
3. As shown in Figure 4(c), the weight data is changed so that the calculation can cover all the feature data and weight data of the sub-block, and all the data of the 3×3 convolution kernel on *n* channels and the entire feature data are calculated. The result of multiplying the feature data corresponding to the 9-weight data of the 3×3 convolution kernel and accumulating in the channel direction.
4. The next *N* channel sub-block is taken along the channel direction to repeat the abovementioned calculation, and the result is accumulated to output the characteristic data.

The maximum pooling calculation is shown in Figure 5. The feature data is divided into multiple *n* × *n* sub-blocks along the length and width, and the maximum value is taken in each sub-block. The length and width of the output feature data are the original feature data lengths. And the width of 1/*n*.

Pooling is an operation used to reduce the size of data.

As shown in Figure 6, to improve the computational efficiency of the pooling module, this paper designs two subfunctions, horizontal pooling and vertical pooling, and uses pipeline parallel calculation to obtain the output results. At the same time, multichannel parallel acceleration is performed on each subfunction.

Assuming that the input feature data is pooled with the maximum value of *n* × *n* and the step size is also *n*, the specific calculation process is as follows:

1. As shown in Figure 6(a), the input feature enters the horizontal pooling module, the first data is compared with the subsequent input *n* − 1 data, and the maximum value is recorded. Take the input *n* data as a group, and repeat the abovementioned operations to obtain the result of horizontal pooling. Currently, the height of the intermediate data remains unchanged, and the width is 1/*n* of the original width.
2. As shown in Figure 6(b), first record the first *W*_out_ data of the intermediate feature input, and compare the *n* − 1 sets of *W*_out_ data input later with the first set of data at the corresponding positions to obtain the maximum value, and output the result. Take the input *n* groups of *W*_out_ data as a group.

## 4. Results and Discussion

The experiment in this paper is based on the three typical datasets of MHEALTH, WHARF, and USCHAD in the UCI_HAR dataset. These three datasets based on wearable devices are represented in the field of human behavior recognition and can reflect the overall performance of this method. To better illustrate the advantages of the method in this paper, experiments were also carried out on two relatively new datasets, the Stanford-ECM Dataset and DATAEGO [24, 25]. Among them, the Stanford-ECM Dataset was published in 2017. The DATAEGO dataset was made publicly available in 2018. Since the dataset may have problems such as unbalanced sample distribution, and these problems may cause overfitting of the model, it is necessary to prove through experiments whether the improvement in model performance is caused by overfitting. This paper also conducts experiments based on the dataset of the Stanford-ECM Dataset and analyzes the reasons for its performance improvement. To verify the versatility of the method, this paper also uses the network in the classification part of the zero-sample learning task. The semantic relationship parameters between the visible class and the unknown class and the prototype features of the visible class are synthesized as the virtual prototype features of the unknown class. The input and output of the network model are the semantic attributes of each category. The category is determined according to the semantic attributes. Furthermore, this is compared with the method proposed by Chen et al. to verify the performance of the algorithm in this paper [26].

### 4.1. Experimental Evaluation Index

In the experiment of this paper, three evaluation indicators are used, namely, precision *A*, recall rate *R*, and *F*_1_ value. In the field of machine learning, *A* is the most common evaluation index, which indicates how many of all samples that the model judges to be positive are true positive samples, which is as follows:

(19) $$\begin{array}{c} A=\frac{\text{TP}+\text{TN}}{\text{TP}+\text{TN}+\text{FP}+\text{FN}}, \end{array}$$

where TP defines a real example, which means that the positive sample is predicted to be the number of samples in the positive class; TN presents a true negative example, which shows that the negative class sample is predicted to be the number of samples in the negative class; FP describes a false positive example, which describes that the positive class sample is predicted to be the number of samples that are predicted to be negative; FN defines a false negative, which explains the number of samples that are predicted to be positive. *R*, known as recall rate, which indicates how many positive samples are judged by the model as positive samples, is also one of the common evaluation indicators in the field of machine learning. Its calculation method is as follows:

(20) $$\begin{array}{c} \text{R}=\frac{\text{TP}}{\text{TP}+\text{FP}}. \end{array}$$

The function of the *F*_1_ value is to consider both *A* and R when evaluating the model and balancing precision and recall. It is also one of the commonly used evaluation indicators. The calculation method is as follows:

(21) $$\begin{array}{c} F_{1}=\frac{2\times A\times R}{A+R}. \end{array}$$

### 4.2. The Process of Sample Generation and the Division of Datasets

For sensor data, samples are obtained by sliding on the original data by setting a fixed time window. There are two ways for the time window to slide on the original data: one is to slide without overlap and the other is to slide with half overlap. The two sample generation methods have their advantages and disadvantages. Among them, the main advantages of generating samples in a nonoverlapping manner are that there is no overlap between the samples and that the experimental results will not cause deviation, but the number of samples generated in this way will be relatively small. With half overlap, the advantage of the method of generating samples is that it can generate as many samples as possible, but its disadvantage is that overlap will bring high deviations, resulting in better results than actual. When training the model, the dataset needs to be divided into a training set, a validation set, and a test set. Since the three datasets used in this paper have user information, cross-validation is used to train the model in the process of training the model. That is, one user data is reserved for model verification in each training, and the data of other users is used for the model verification train. Doing so means that each user's data will be used as a validation set, which means that multiple experiments are required. Considering that there may be situations where the quality of the data collected by the user is low or beyond expectations, the maximum and minimum values are removed in the final evaluation of the model, and the average value is taken to evaluate the performance of the model more comprehensively.

### 4.3. Experiment and Result Analysis

This paper conducts experiments on the five abovementioned datasets and compares different methods. To ensure comparability between the methods, this paper sets the same experimental conditions and experimental end conditions during the training model. That is, the training model process ends when the loss value is less than or equal to 0.2 or after 200 iterations of training are completed. This paper uses Adadelta as the optimizer, and the Softmax classifier as the classifier. The learning rate of the model is 0.001, and the maximum number of iterations is 200.

It can be seen from Table 1 that compared with the method of Chen et al., the method in this paper has obvious advantages in the three commonly used evaluation indicators. This fully illustrates the necessity of data fusion and the reasonable setting of convolution kernels in data feature extraction for such tasks. The method in this paper has achieved better results on the MHEALTH dataset, and the accuracy reaches 94.08%, which is 2.21% higher than Chen et al.'s method, which is enough to prove the advantage of this method. In addition, the method in this paper also has obvious advantages in the WHARF dataset and the USCHAD dataset, but the effect is not significantly improved in the MHEALTH dataset. The reason is that the dataset is collected in different ways. The MHEALTH dataset has strict data during the collection process. The collection standard regulates the collection action. However, the WHARF dataset and the USCHAD dataset did not develop such strict collection standards during the collection process.

Figure 7 shows the experimental results of the two methods on the Stanford-ECM Dataset. It can be seen from Figure 7 that the method in this paper has achieved better results in 8 categories. With the same results of the method, 5 categories have achieved slightly worse results. However, the overall performance is still significantly improved, indicating that the performance improvement is not caused by the data distribution but the function of the method itself.

## 5. Conclusions

This paper proposes a method for feature extraction of wearable sensor data based on CNN. This method first uses a Kalman filter to fuse the data to obtain a preliminary state estimation, and then uses CNN to recognize human behavior and obtain the corresponding behavior set. This paper conducts experiments on five datasets. The experimental results show that this paper can extract data features at multiple scales while fully maintaining data independence and can effectively extract corresponding feature data. In addition, the method in this paper has strong generalization ability and can adapt to different learning tasks. At present, wearable devices are mainly smart watches and bracelets, concentrated in medical and health, outdoor sports, audio-visual entertainment, and other fields. With the intensification of society's aging phenomenon, the wearable device market will usher in tremendous development in areas where health is the appeal. In the future, the accurate extraction of data characteristics of wearable sensors can be used to analyze users' various behaviors, the health index, and other data, which also provides strong support for disease prevention and treatment, health monitoring, and other aspects. At the same time, the accurate extraction of wearable sensor data features can complete various tasks such as object detection, face recognition, and image analysis, bringing a brand new experience to users. The accurate extraction of data features of wearable sensors can provide humans with more accurate and reliable basic datasets. Through these datasets, more intelligent and digital behavior parameters can be provided for artificial intelligence and help the development of artificial intelligence.

## Figures and Tables

**Figure 1:** Data feature extraction process based on wearable sensors.

**Figure 2:** Flowchart of the data fusion algorithm based on the extended Kalman filter.

**Figure 3:** Convolution calculation module.

**Figure 4:** Convolution operation flowchart.

**Figure 5:** Max pooling calculation.

**Figure 6:** Pooling flowchart.

**Figure 7:** Experimental results based on the dataset of the Stanford-ECM Dataset.

**Table 1:** Experimental results of two methods.

Data set	Method	*A* (%)	R (%)	*F*_1_ (%)
HEALTH	Chen et al.	98.1	91.3	90.1
	This paper	94.	94.1	93.1

WHARF	Chen et al.	67.1	42.9	42.6
	This paper	68.7	44.1	43.8

USTAD	Chen et al.	78.8	74.6	71.4
	This paper	79.6	76.8	73.2

Stanford-ECM Dataset	Chen et al.	92.3	88.1	88.8
	This paper	93.7	88.8	90.1

DATAEGO	Chen et al.	55.2	43.8	43.0
	This paper	58.2	45.7	44.7

## Data Availability

The datasets used and/or analyzed during the current study are available from the author on reasonable request.
